# Identification and Validation of Invasion-Related Molecular Subtypes and Prognostic Features for Cervical Cancer

This article has been retracted.

**DOI:** 10.1155/2022/1902289

**Published:** 2022-03-18

**Authors:** Xingling Wang, Jing Wang, Mingxin Yu

**Affiliations:** Department of Gynecology, Cancer Hospital of China Medical University, Liaoning Cancer Hospital & Institute, No. 44 Xiaoheyan Road, Dadong District, Shenyang, 110042 Liaoning Province, China

## Abstract

**Background:**

As one of the main causes leading to female cancer deaths, cervical cancer shows malignant features of local infiltration and invasion into adjacent organs and tissues. This study was designed to categorize novel molecular subtypes according to cervical cancer invasion and screen reliable prognostic markers.

**Methods:**

Invasion-related gene sets and expression profiles of invasion-related genes were collected from the CancerSEA database and The Cancer Genome Atlas (TCGA), respectively. Samples were clustered by nonnegative matrix factorization (NMF) to obtain different molecular subgroups, immune microenvironment characteristics of which were further systematically compared. Limma was employed to screen differentially expressed gene sets in different subtypes, followed by Lasso analysis for dimension reduction. Multivariate and univariate Cox regression analysis was performed to determine prognostic characteristics. The Kaplan-Meier test showed the prognostic differences of patients with different risks. Additionally, receiver operating characteristic (ROC) curves were applied to validate the prognostic model performance. A nomogram model was developed using clinical and prognostic characteristics of cervical cancer, and its prediction accuracy was reflected by calibration curve.

**Results:**

This study filtered 19 invasion-related genes with prognosis significance in cervical cancer and 2 molecular subtypes (C1, C2). Specifically, the C1 subtype had an unfavorable prognosis, which was associated with the activation of the TGF-beta signaling pathway, focal adhesion, and PI3K-Akt signaling pathway. 875 differentially expressed genes were screened, and 8 key genes were finally retained by the dimension reduction analysis. An 8-gene signature was established as an independent factor predictive of the prognosis of cervical cancer. The signature performance was even stronger when combined with N stage.

**Conclusion:**

Based on invasion-related genes, the present study categorized two cervical cancer subtypes with distinct TME characteristics and established an 8-gene marker that can accurately and independently predict the prognosis of cervical cancer.

## 1. Introduction

Cervical cancer has been reported as the second major contributor of cancer fatalities in women between the ages of 20 and 39 [1]. In the past 30 years, increasing awareness of the disease and advancement in medical measures including prevention, screening, and improved treatment and the occurrence, mortality, and disability-adjusted life years (DALYs) are all decreasing progressively [2, 3]. Nevertheless, patients' prognosis having metastatic and recurrent cervical cancer is unfavorable, and the clinical treatment faces a great challenge [2]. Therefore, it is vital to effectively anticipate the patients' prognosis in order to provide guidance in the formulation of clinical therapeutic plans.

Cervical cancer is usually histologically classified into different subtypes, including squamous cell carcinoma occurring in the outer cervix (accounting for about 75% of invasive cervical cancer cases), adenocarcinoma originating from the cervical canal, and less common adenosquamous, serous papilla, and clear cell carcinoma of the cervix and small cell or neuroendocrine. Cervical cancer is a heterogeneous cancer showing heterogeneity also in other aspects, such as molecular characteristics [4], metabolism [5], invasive risk [6], local microenvironments [7], and responses to treatment [8]. Hence, subtype classification related to these factors is critical to the treatment and prognosis of patients.

The formation of large-scale gene expression datasets along with the emergence of high-throughput gene detection technologies has made it possible to classify patients in a more precise manner and identify the key molecular characteristics combined with clinical characteristics for a better design of personalized treatment plans for patients [9]. As invasion is one of the important clinical parameters affecting the prognosis of patients with cervical cancer, this study developed a subtype classification of patients with cervical cancer according to the cervical cancer invasion-related genes. We carried out hierarchical clustering of cervical cancer according to invasion-related genes to develop subtype categorization of patients with cervical cancer. The characteristics of subtypes in the tumor microenvironment (TME) were also discussed. Next, based on subtype classification, the prognosis prediction model of cervical cancer was determined using machine learning methods, and its validity and reliability were verified in internal and external validation cohorts. The new classification of cervical cancer may guide clinical decision-making for personalized treatment of cervical cancer patients.

## 2. Materials and Methods

### 2.1. Acquisition of Sample Raw Data

RNA transcription data along with clinical features of two cervical cancer cohorts were, respectively, acquired from The Cancer Genome Atlas (TCGA) (https://portal.gdc.cancer.gov/) and Gene Expression Omnibus (GEO) databases. 291 samples in TCGA were classified into the internal training set (*n* = 146) and internal test set (*n* = 145), while the other 300 samples in GSE44001 [10] were also taken as the verification set. Samples from both cohorts had survival status data and overall survival (OS). CancerSea [11] was employed to obtain 97 invasion-related genes. The clinical information of datasets is shown in Table 1.

### 2.2. Consensus Clustering Analysis

With respect to the 97 invasion-related genes (Supplementary Table 1), we conducted a univariate Cox analysis to screen prognostic genes of cervical cancer. Based on cervical prognostic genes, the nonnegative matrix factorization (NMF) clustering approach was employed in the clustering of cervical cancer samples. The best cluster number was calculated using cophenetic, suspension, and silhouette. Clinical characteristics, including the age of survival status; N, T, M, and AJCC stages and grade; and survival of specific molecular subgroups were compared in different clusters to assess the reproducibility of invasion gene-based molecular subgroup prediction system.

### 2.3. Tumor Microenvironment (TME) Analysis between Clusters

ESTIMATE [12] in the R software package was employed to predict immune, stromal, and ESTIMATE scores of different clusters to indicate the degree of infiltrating matrix as well as immune cells in TME and tumor purity. The score of 38 TME cells was determined according to MCP-Counter [13] and the ssGSEA [14] of the GSVA package.

### 2.4. Screening and Enrichment Analysis of Differentially Expressed Genes (DEGs)

Package Limma [15] was employed to examine gene expression differences between different clusters. FDR < 0.05 and | | FC > 1.5 DEGs were considered to be significant. Significant DEGs were screened for KEGG and GO enrichment analysis in the R software packageWebGestalTR [16].

### 2.5. Establishment of Prognostic Risk Scores according to DEGs between Clusters

R software package survival coxph function in TCGA intertrain set was utilized to conduct univariate Cox regression analysis so as to detect prognosis-related invasive genes with *P* < 0.01. Lasso and multivariate Cox regression were utilized to establish a prognostic model. The components of the model were further simplified by StepAIC in the MASS package. The overall survival (OS) was estimated utilizing the log-rank test as well as the Kaplan-Meier survival curves. The R package “timeROC” [17] was employed to draw the receiver operating characteristic (ROC) curve, and the area under the curve (AUC) of the OS over one, three, and five years was calculated using “livingROC.” Both multivariate and univariate Cox regression analyses were conducted to determine if the predictive performance of the risk score was influenced by additional clinical variables.

### 2.6. Subgroup Survival Analysis

Samples of cervical cancer in TCGA were classified into different subgroups based on their age, T stage, AJCC stage, N stage, M stage, and grade. Each set of patients was further categorized into high- and low-risk groups. A survival study was carried out so as to examine the prognostic differences between the low- and high-risk groups.

### 2.7. Construction of a Nomogram

Two independent prognostic indicators, risk score and N stage, were integrated to create a nomogram using the R package “RMS.” For the purpose of determining the correlation between anticipated survival by the nomogram and actual survival, calibration plots were created. The net benefit was determined using decision curve analysis (DCA) on both the clinical features and combination models.

### 2.8. Statistical Analysis

All statistical analysis of this project was undertaken in R package (version 3.6.3). The Wilcoxon test was utilized to detect statistical differences between two groups of variables, while statistical differences between over 2 groups of variables were analyzed by the Kruskal test. If there was no special explanation, the default *P* < 0.05 was employed to assess statistical significance.

## 3. Results

### 3.1. Identification of Two Subclasses of Cervical Cancer

The whole analysis process is illustrated in Figure S1A. The univariate Cox regression analysis revealed that 19 of the 97 invasion-related genes were associated with the OS of cervical cancer. Unsupervised NMF clustering was used to identify two subgroups (Supplementary Table 2), cluster 1 (C1) and cluster 2 (C2), based on 19 invasion-related genes (Figures 1(a) and 1(b)). A heat map was drawn to examine the expression differences of the nineteen genes between two clusters, and more than three-quarters of the genes were low-expressed in C2 and overexpressed in C1 (Figure 1(c)). Kaplan-Meier curves showed that patients in C2 had a significant survival advantage over those in C1 (Figure 1(d)). We compared the distribution of HPV in C1 and C2 subtypes. Although there was no significant difference between the two groups (*P* = 0.35), a higher proportion of HPV in the C2 subtype can be observed (Figure S1B).

### 3.2. TME Features of Cervical Cancer Subclasses

We applied GSEA to examine the differences in pathways between the two subclasses and found that focal adhesion, the signaling pathway of TGF-*β* in cancer, and signaling pathway of Wnt showed an increase in GSEA score in the C1 group (Figure 2(a)). ESTIMATE predicted the relationship between cervical cancer subclasses and TME characteristics and demonstrated that immune, stromal, and ESTIMATE scores were statistically different for patients in C1 and C2. ESTIMATE score and stromal score of patients in C1 were greater compared to those in C2, and immune score was higher for C2 (Figure 2(b)). Such results indicated more matrix components in the TME of C1 patients and a higher proportion of immune components in the TME of C2 patients. Immune scores of 10 TME cells for C1 and C2 as indicated by MCP-Counter calculation demonstrated that among the 7 TME cells showing statistical differences between C1 and C2, T cells, cytotoxic lymphocytes, CD8 T cells, and myeloid dendritic cells had a greater immune score in C2 patients, while matrix cells, including fibroblasts, and colorectal cells were higher in the TME of C1 patients. Provide further evidence for the above inference (Figure 2(c)). From ssGSEA, it was found that there were 11 types of TME cells with different immune scores between C1 and C2 (Figure 2(d)).

### 3.3. The Clinicopathologic Features of the Molecular Subtypes

By studying the clinicopathologic features of the two molecular types, we found that C1 was associated with the dead event of the two molecular subtypes (Figure 3(a)). There was no substantial difference in the distribution of the age between the 2 molecular subgroups (Figure 3(b)). In terms of N stage, T stage, AJCC stage, M stage, and grade, C1 was associated with a more advanced cancer stage than C2 but without a statistical difference (Figures 3(c)–3(g)). Then, the clustering typing results were compared with the molecular subtype previously reported [18], and the comparison results showed that there was a significant correlation between our clustering typing results and previous typing results (Figures 3(h) and 3(i)).

### 3.4. DEGs and Functions Between C1 and C2 Subtypes

According to the difference analysis, 857 DEGs were identified in the C1 and C2 samples, 793 out of the 857 DEGs were overexpressed, and the rest 82 were underexpressed (Figure 4(a)). The heat map of 100 DEGs in between C1 and C2 is intersected and illustrated in Figure 4(b). For all the DEGs, the enrichment pathway was mostly correlated with an extracellular matrix organization, ossification, and epithelial cell proliferation (Figure 4(c)). KEGG analysis illustrated the enrichment of DEGs in several pathways associated with tumor genesis, progression, and prognosis, including cell adhesion molecules, TGF-*β* signaling pathway, focal adhesion, proteoglycans in cancer, ECM–receptor interaction, PI3K–Akt signaling pathway, human papillomavirus infection, and cytokine–cytokine receptor interaction (Figure 4(d)).

### 3.5. Development of a Prognostic Model for Cervical Cancer Patients according to DEGs between C1 and C2 Subgroups

Using TCGA intertrain set, univariate Cox analysis excluded DEGs without significant correlation with OS, and the remaining 24 DEGs were regarded as risk indicators for the prognosis of patients with cervical cancer. Lasso Cox regression analysis results are shown in Figure 5(a), and a 14-gene combination was generated. StepAIC further simplified the 14-gene combination to an 8-gene combination. The following risk scores were obtained for the patients: risk score = 0.16∗ALG1L − 0.153∗ARMCX1 − 0.519∗ASCL2 − 0.104∗CST6 + 0.193∗CXCL2 − 0.105∗DES + 0.418∗OPN3 − 1.995∗SERPINF1. AlG1L, AsCl2, and DES were protective factors, whereas ARMCX1 and CST6 were risk factors (Figure S2). According to the risk score formula, each sample was risk-scored accordingly and was assigned to different risk groups. The number of patients who died steadily climbed as the risk score increased (Figure 5(b)). Individuals at high risk of death had a considerably shorter life expectancy than patients at low risk (Figure 5(c)). The predictive capacity of the risk score was further examined using the ROC curve. The one-, three-, and five-year OS as demonstrated by the AUCs of the ROC curves was 0.89, 0.91, and 0.89, respectively (Figure 5(d)), showing high sensitivity and specificity of the score in the prognostic assessment of cervical cancer cases in TCGA intertrain set. Further, we compared the differences of 8 prognostic genes in the two subtypes. It can be observed that ARMCX1, CST6, CXCL2, DES, OPN3, and SERPINF1 are significantly overexpressed in C1 and significantly underexpressed in ALG1L and ASCL2 (Figure S3A). Interestingly, ALG1L and CST6 of the eight prognostic genes were significantly overexpressed in HPV-positive patients (Figure S3B). In addition, we also observed that CXCL2 was significantly overexpressed in tumor samples (Figure S3C). We also compared the difference of risk score between HPV-positive and HPV-negative patients. Unfortunately, no significant difference was observed, which may be related to the small number of HPV-negative samples (Figure S3D).

### 3.6. Verification of a Prognostic Model for Cervical Cancer Patients according to DEGs between C1 and C2 Subtypes

We further validated the prognostic model for cervical cancer patients in other cohort groups, including TCGA intertest set (*n* = 145), TCGA-CESC cohort, and the GSE44001 cohort. Due to the crossplatform batch effect, patients in each cohort were arranged in an ascending order of standardized risk score and classified into low- and high-risk groups based on the threshold point of 0 (Figures 6(a)–6(c)). The high-risk group displayed a considerably worse OS as opposed to that of the low-risk group in all three validation queues (Figures 6(d), 6(f), and 6(h)). Then, the ROC curve analysis was undertaken, and the AUCs of the ROC curves for one-, three-, and five-year OS were 0.52, 0.7, and 0.76 in TCGA internal test set (Figure 6(e)). In TCGA-CESC cohort (*n* = 291), the AUCs of the ROC curves for one-, three-, and five-year OS reached 0.65, 0.8, and 0.82, respectively (Figure 6(g)). For the cohorts of GSE44001, the AUC value of ROC for one-, three-, and five-year OS were 0.8, 0.66, and 0.66 (Figure 6(i)). These verification findings illustrated that the risk model constructed in the present research was highly effective in anticipating the prognosis of patients with cervical cancer.

### 3.7. Risk Score Independently Stood as a Prognostic Indicator for Cervical Cancer Patients

We assessed the prognostic value of the risk score model with diverse clinicopathological characteristics, and all TCGA-related patients were categorized into two groups based on different clinical factors, including T stage, age, N stage, AJCC stage, M stage, and grade. Following that, patients in various subgroups were additionally classified into low- and high-risk groups. In the subgroup of age > 45 (Figure 7(a)), age = 45 (Figure 7(b)), T1-T2 stage (Figure 7(c)), N0 stage (Figure 7(e)), N1 stage (Figure 7(f)), M0 stage (Figure 7(g)), stages I-II (Figure 7(i)), stages III-IV (Figure 7(j)), G1-G2 (Figure 7(k)), and G3 (Figure 7(l)), high-risk score patients presented a substantially shorter OS compared to those with low-risk scores. However, in the T3-T4 stage (Figure 7(d)) and 7M stage (Figure 7(h)) subgroups, there was no strong association between OS and risk score of cervical cancer patients. Univariate Cox analysis of clinical variables in TCGA demonstrated that risk score, N stage, AJCC stage, M stage, and T stage had a significant correlation with OS of cervical cancer (Figure 7(m)). After adjusting the confounding variables, multivariate Cox analysis indicated that only N stages and risk score independently served as prognostic indicators for cervical cancer (Figure 7(n)).

### 3.8. Development of a Prognostic Anticipation Nomogram for Cervical Cancer

A nomogram was developed according to the independent prognostic factor risk score and N stage of cervical cancer. Every prognostic factor was assigned a score, and the total of the two predictive score factors was employed to anticipate the 1-, 3-, and 5-year rates of survival of patients with cervical cancer, with a greater total score indicating a poor prognosis (Figure 8(a)). To determine if the nomogram is clinically applicable, the DCA results showed that the combined model had a net benefit in anticipating OS and demonstrated a greater clinical benefit compared to the risk scoring model (Figure 8(b)). The 1-, 3-, and 5-year OS predicted by the calibration curve was close to the results of the ideal model, suggesting that the histogram had a strong prediction ability and high accuracy (Figure 8(c)).

## 4. Discussion

Cancer cells seed secondary tumors at distant sites through invasion mechanism [19]. Cervical cancer is a tumor with invasion heterogeneity [6]. In this study, we determined patients belonging to two types of subclasses. C1 of cervical cancer showed poor prognosis and had a higher stromal score and ESTIMATE score based on invasion-related genes. In addition, stromal cells, including fibroblasts and endothelial cells, were higher in the TME of C1 patients, suggesting more matrix components in the TME of C1 patients. C2 patients showed a significantly better prognosis and higher immune score. Moreover, immune components, including CD8 T cells, T cells, cytotoxic lymphocytes, and myeloid dendritic cells, also scored higher in C2 patients, indicating that C2 patients showed a larger percentage of immunological components in the TME.

The development in bioinformatics, particularly in high-throughput sequencing technology, has made it possible to study the underlying mechanisms of cancer at the transcriptome level. Bioinformatics tools have been increasingly applied to develop efficient signatures that may be used to improve prognosis and uncover the underlying mechanisms of various cancers [20]. Zhang et al. identified three prostate cancer subtypes by integrative bioinformatics analysis and developed a 12-gene risk prediction model [21]. In LUAD, a study established a new prognostic gene expression signature based on genes related to DNA repair and identified two distinct molecular subgroups having different clinical characteristics [22]. In gastric cancer, bioinformatics tools were employed to identify two subgroups having different immune and clinical features, and a risk scoring model based on seven genes was created according to different expression patterns among subtypes [23]. After identifying the characteristics of cervical cancer subtypes, we analyzed the DEGs between subtypes and constructed a risk anticipation model based on 8 prognostic DEGs, which divided cervical cancer patients into low- and high-risk groups. The effectiveness of the risk score model was also verified in internal and external cohorts. When patients with cervical cancer were regrouped according to different clinicopathologic features, the risk score model also showed accurate and independent predictive power.

For the genes in the risk model, in addition to CXCL2 [24] and DES [25], the other six genes were associated with a variety of cancers other than cervical cancer. ALG1L is a potential biomarker for hepatocellular carcinoma [26]; ARMCX 1 participates in multiple cellular functions in gastric cancer, such as migration, cell proliferation, and invasion, as well as cytoskeleton structure destruction [27]. The ASCL2 expression is positively correlated with breast tumor size, lymphatic metastasis, and active tumor cell growth and can be used as a marker to evaluate the tumor recurrence risk [28]. Also, cancer-derived soluble CST6 in breast cancer could inhibit the spread of cancer cells [29]. OPN3 promoted cancer cell metastasis and epithelial-mesenchymal transformation of lung adenocarcinoma [30]. SERPINF1 has been identified as associated with ovarian cancer prognosis and can serve as a biomarker to monitor patients' survival with ovarian cancers [31]. Here, the combination of these 8 genes was also considered as a prognostic factor for cervical cancer. Combining the clinical factor N stage with the prognostic model can bring benefits to the prognosis improvement for cervical cancer patients.

## 5. Conclusion

Taken together, the present study found two distinct molecular subgroups based on invasion-related genes with different survival outcomes and TME characteristics. On the basis of DEGs between the two subtypes, a prognostic risk model for cervical cancer was created and was also internally and externally validated with good accuracy and independence in anticipating patients' clinical outcomes. Our finding provides new data for the further understanding of cervical cancer patients' treatment and prognosis.

## Figures and Tables

**Figure 1:** Identification of two subclasses of cervical cancer. (a) Clustering display of the subclasses. (b) Estimation of the factorization rank (2 to 10; *x*-axis) using the residual sum of squares (rss), cophenetic, and dispersion coefficients (*y*-axis). Cophenetic correlation, dispersion analysis, and residual sum of squares (rss). (c) Heat maps showed differences in 19 invasion-related gene expressions between C1 and C2. (d) Kaplan-Meier curves revealed the patients' OS in C1 and C2.

**Figure 2:** TME features of cervical cancer subclasses. (a) GSEA analyzed the differences in physiological pathways between the C1 and C2. (b) ESTIMATE predicted the relationship between cervical cancer subclasses and TME characteristics. (c) Immune scores of 10 TME cells between C1 and C2 were obtained by MCP-Counter. (d) ssGSEA analyzed the immune score of 28 TME cells between the patients with exhibited C1 and C2.

**Figure 3:** The clinicopathologic features of the molecular subtypes. (a–g) Patients were classified according to clinical characteristics, such as survival events, T stage, age, N stage, AJCC stage, M stage, and grade. (h) Sankey plot showed consistency between the classifier based on 19 invasive-related genes and the results of existing cervical cancer classifications. (i) Correlation between classifiers based on 19 invasion-related genes and results of existing cervical cancer classifications.

**Figure 4:** DEGs and their functions between two molecular subtypes. (a) Differential expression analysis between C1 and C2 samples. (b) The heat map showed the TOP50 genes with high and low expression differences between samples in C1 and C2. (c) GO analysis of DEGs between C1 and C2 samples, such as biological processes, molecular function, and cellular component. (d) DEG comparison between C1 and C2 samples using KEGG.

**Figure 5:** Development of a prognostic model for cervical cancer patients according to DEGs between C1 and C2 subtypes. (a) Lasso analysis to determine the optimal genes for the model. (b) TCGA internal training set patients were arranged from the lowest to the highest risk score and heat map of expression of 8 genes in the model. (c) Kaplan-Meier curves of patients having different risk levels in TCGA internal training set. (d) ROC curves for 1-, 3-, and 5-year OS.

**Figure 6:** Verification of prognostic signature of cervical cancer patients based on DEGs between C1 and C2 subtypes. (a) TCGA internal test set patients were ranked from the lowest to the largest risk score and heat map of expression of 8 genes in the model. (b) Patients with cervical cancer in TCGA-CESC cohort were listed in an ascending order of risk score as well as the heat map of expression of 8 genes in the model. (c) All patients in the GSE44001 cohort were listed in an ascending order of risk score and heat map of gene expression in the model. (d) The log-rank test was utilized to evaluate the statistical significance of the difference between the high- and low-risk groups in TCGA internal test set cohort. (e) The ROC curve for1-, 3-, and 5-year OS in TCGA internal test set. (f) In TCGA-CESC cohort, Kaplan-Meier curves for survival analysis. (g) The AUCs of the ROC curves for 1-, 3-, and 5-year OS in TCGA-CESC cohort. (h) The Kaplan-Meier curve of different risk groups. (i) ROC curves in the GSE44001 cohort and AUC were applied to determine the accuracy of the risk model.

**Figure 7:** Prognostic significance and independence of risk scoring models with different clinicopathologic features. In TCGA-CESC cohort, prognostic differences between patients at low risk and high risk in different subtypes, including (a) age > 45, (b) age = 45, (c) T1-T2 stage, (d) T3-T4 stage, (e) N0 stage, (f) N1 stage, (g) M0 stage, (I) stages I-II, (j) stages III-IV, (k) G1-G2, and (l) G3. Univariate Cox analysis (m) and multivariate Cox analysis (n) determined that N stage and risk score were an independent prognostic indicator among clinical factors in TCGA-CESC cohort.

**Figure 8:** Construction of a prognostic prediction nomogram for cervical cancer. (a) Nomogram based on risk score and N stage. (b) Calibration chart for internal validation of the nomogram, and the dotted line represents the ideal calibration line. (c) DCA curve of the nomograms for 1-, 3-, and 5-year OS.

**Table 1:** Clinical information of cervical cancer patients in TCGA and GEO databases.

Clinical features	TCGA-CESC	GSE44001
OS		
0	220	262
1	71	38
T stage		
T1	137	
T2	67	
T3	16	
T4	10	
TX	61	
N stage		
N0	128	
N1	55	
NX	108	
M stage		
M0	107	
M1	10	
MX	174	
Stage		
I	159	
II	64	
III	41	
IV	21	
X	6	
Grade		
G1	18	
G2	129	
G3	116	
G4	1	
GX	27	
Age		
≤45	139	
>45	152	

## Data Availability

The data used to support the findings of this study are included within the article.

## Supplementary Materials

Supplementary 1 Supplementary Figure S1 A: overview of the analysis process of this study. B: HPV distribution in two molecular subtypes.

Supplementary 2 Supplementary Figure S2: survival curves of cervical cancer patients grouped according to the expression of each gene in the risk score model.

Supplementary 3 Supplementary Figure S3: the expression difference of 8 genes. A: expression differences of 8 genes in two molecular subtypes. B: the expression difference of 8 genes in HPV-positive and HPV-negative patients. C: the expression of 8 genes was different between cancer and adjacent cancer. D: differential distribution of risk score in HPV-positive and HPV-negative patients.

Supplementary 4 Supplementary Table 1: list of invasion-related genes.

Supplementary 5 Supplementary Table 2: molecular subtype information of each sample in TCGA dataset.
